The article "Vitamin D Status and All-Cause Mortality in Patients With Type 2 Diabetes in China" was published in 2022. Journal: Front Endocrinol (Lausanne).

# Vitamin D Status and All-Cause Mortality in Patients With Type 2 Diabetes in China

**DOI:** 10.3389/fendo.2022.794947

**Published:** 2022-03-04

**Authors:** Yuxin Fan, Li Ding, Yalan Zhang, Hua Shu, Qing He, Jingqiu Cui, Gang Hu, Ming Liu

**Affiliations:** ^1^ Department of Endocrinology and Metabolism, Tianjin Medical University General Hospital, Tianjin, China; ^2^ Chronic Disease Epidemiology Laboratory, Pennington Biomedical Research Center, Baton Rouge, LA, United States

**Keywords:** vitamin D, 25-OH vitamin D, type 2 diabetes, all-cause mortality, 1,25-(OH)2D3

## Abstract

**Objective:**

To assess the association between vitamin D status and all-cause mortality among type 2 diabetes patients.

**Research Design and Methods:**

We prospectively followed 1,291 participants with type 2 diabetes aged 20–80 years during 2013–2018. Cox proportional hazard regression models were used to estimate the association between different vitamin D status and all-cause mortality risk among hospitalized patients with type 2 diabetes.

**Results:**

During a median follow-up of 4.15 years (5,365 person-years in total), 61 cases of death were identified. Multivariable-adjusted hazard ratios (HRs) for all-cause mortality across the quartiles of baseline circulating 25-hydroxy vitamin D (25-OH vitamin D) were 2.70 [95% confidence interval (CI) 1.12–6.54], 1.00, 1.39 (95% CI 0.53–3.65), 2.31 (95% CI 0.96–5.54), respectively. Multivariable-adjusted HRs for all-cause mortality by different groups of baseline 25-OH vitamin D concentrations (<25, 25–49, 50–100, and ≥100 nmol/L) were 1.31 (95% CI 0.58–2.96), 0.94 (95% CI 0.47–1.87), 1.00, and 3.58 (95% CI 1.43–8.98), respectively.

**Conclusions:**

Very low or high concentrations of vitamin D may be associated with a higher risk of all-cause mortality among patients with type 2 diabetes.

## Introduction

The prevalence of type 2 diabetes has already reached up to 10.9% (1) in Chinese adults and is projected to reach over 500 million by 2030, implicating significant burdens of morbidity and mortality (2). Moreover, diabetes is one of the most leading causes of death and is ranked 20th in China in 2017 (3). The risk of mortality among people with type 2 diabetes is significantly higher than that among the general population (4). Therefore, identifying individuals who are at a relatively high risk of death among patients with type 2 diabetes is imperative for cost-effective intervention to reduce the associated enormous economic burden.

In recent years, testing vitamin D levels has attracted more and more attention (5). Vitamin D is an essential fat-soluble nutrient with a crucial role in the regulation of calcium-phosphate metabolism and is obtained from dietary intake and sunlight being biologically inert. Vitamin D is firstly hydroxylated by the 25-hydroxylase to 25-hydroxy vitamin D (25-OH vitamin D) in the liver and then further hydroxylated in the kidney by the 25(OH)D-1α-OHase to 1,25-(OH)_2_ Vitamin D, which is a biologically active form of vitamin D (6, 7). However, serum circulating 25-OH vitamin D is the main storage form of vitamin D and its half-life period is 2–3 weeks, which is much longer than that of 1,25-(OH)_2_D, thus 25-OH vitamin D is considered as the biomarker to determine the serum circulating vitamin D level according to the Endocrine Society Clinical Practice Guidelines (8). Growing epidemiological evidence has indicated that vitamin D deficiency was associated with increased risks of incident diabetes and cardiovascular disease, and also all-cause mortality (9–13). However, a study indicated that vitamin D levels were inversely associated with the risk of death in a general older men population (14). To date, clinical data on vitamin D status, especially for a high concentration of vitamin D on all-cause mortality, are still controversial. The results from the National Health and Nutrition Examination Survey (NHANES) III during a 9-year follow-up have suggested a reverse J-shaped relationship between circulating 25-OH vitamin D levels and the risk of all-cause mortality (15). Several studies have shown that subjects with diabetes had lower serum concentrations of vitamin D (16). However, very few studies have evaluated the association between vitamin D and all-cause mortality in patients with type 2 diabetes. Thus, in the present study, we used 25-OH vitamin D as an indicator to assess the association between circulating vitamin D concentrations and all-cause mortality among patients with type 2 diabetes in China.

## Research Design and Methods

### Study Sample

The present cohort dataset was extracted from the inpatient database of the Department of Endocrinology and Metabolism of Tianjin Medical University General Hospital. We collected all electronic medical records of inpatients with type 2 diabetes at discharge from June 2013 to May 2018 and made telephone follow-ups of the patients. After excluding the subjects with acute illness such as diabetes ketoacidosis or hyperglycemic hyperosmolar status before hospitalization, the study population finally included 1,291 inpatients aged 20–80 years old with baseline measurements of weight, height, blood pressure, 25-OH vitamin D, fasting plasma glucose, low density lipoprotein (LDL) cholesterol, estimated glomerular filtration rate (eGFR), glycated hemoglobin a1c (HbA1c) and high-density lipoprotein (HDL) cholesterol (**Figure 1**). Other 2,504 individuals from the present cohort dataset were not selected due to lack of baseline measurements or loss of follow-up. Compared with those included in the study, the excluded patients were younger (aged 55.5 years versus 57.2 years), had less women (48.3% versus 58.1%) and more smokers (32.9% versus 28.3%). Informed consent of patients was not obtained because the present study was a secondary data analysis, which did not need to include personally identifiable information except for birth date. The study was approved by the Tianjin Medical University General Hospital Institutional Review Board approval number (IRB2020-YX-027-01) and the individual informed consent was waived.

**Figure 1:** Flow chart of identification of the study population.

### Measurements

Information on date of birth, sex, insurance status, age of diabetes diagnosis, smoking status (current smokers and non-smokers), alcohol drinking (current alcohol consumers and non-alcohol consumers), history of chronic diseases (angina, coronary heart disease, or stroke), and use of agents (such as anti-platelet, anti-hypertensive, glucose-lowering agents or cholesterol-lowering drugs) of patients was collected through a standardized electronic inpatient medical record. At admission, trained doctors measured height, weight, and blood pressure using a standard protocol. Standing height was measured to the nearest 0.1 cm using a portable stadiometer. Weight was measured to the nearest 0.1 kg. Height and weight were measured with light clothing and without shoes. Body mass index (BMI) was current weight in kilograms divided by the square of height in meters. Blood pressure was measured two times using a standard mercury sphygmomanometer after 5 min of sitting, and the measurements were averaged. Blood samples were collected after an 8–12-hour overnight fast for all inpatients. Plasma glucose was tested enzymatically by an autoanalyzer (Hitachi Model 7600 analyzer, Hitachi). HbA1c separation and quantification were performed by an HPLC analyzer (HDL-723 G8; Tosoh) with the intra- and interassay coefficients of variation <3%. 25-OH vitamin D was measured by a chemiluminescence immunoassay test using Architect I2000SR analyzer with the intra- and interassay coefficients of variation <4%. LDL cholesterol was measured by the polyvinyl sulfuric acid precipitation method while HDL cholesterol was measured by the chemical precipitation method using appropriate kits (Hitachi 7600 Automatic Biochemistry Analyzer, Hitachi, Tokyo, Japan [from June 2013 to December 2016 and Hitachi 008A Automatic Biochemistry Analyzer, Hitachi, Tokyo, Japan [from January 2017 to May 2018]). eGFR was estimated using the Modification of Diet in Renal Disease (MDRD) (17).

### Vitamin D Deficiency

To date, the definition of vitamin D deficiency has not been universally generalized yet. According to the Institute of Medicine (18) or the Endocrine Society (8) recommendations and published pieces of literature (19, 20), we categorized 25-OH vitamin D levels into four groups: 1) severe vitamin D deficiency (<25.00 nmol/L); 2) vitamin D insufficiency (25–49 nmol/L); 3) vitamin D sufficiency (50–100 nmol/L); and 4) high vitamin D concentrations (>100 nmol/L).

### Definition of Type 2 Diabetes

According to the American Diabetes Association (ADA) guidelines, type 2 diabetes is defined as: 1) self-reported doctors-diagnosed diabetes, or 2) fasting plasma glucose concentrations ≥7.0 mmol/L, or 3) 2-h plasma glucose concentrations ≥11.1 mmol/L, or 4) HbA1c ≥6.5%.

### Prospective Follow-Up

Follow-up data were collected from hospital medical records of readmission or telephone contacts with patients or family members. The primary outcome was all-cause mortality. The duration of follow-up for each patient (person-years) was calculated from the baseline date (the date of first hospitalization) to the date of death, or the date of telephone follow-up.

### Statistical Analysis

We used Chi-square tests and ANOVA test to analyze the prevalence of categorical variables and mean levels of continuous variables across quartiles of plasma 25-OH vitamin D. The Cox proportional hazard regression was used to evaluate the association between baseline circulating 25-OH vitamin D concentrations and the risk of all-cause mortality in patients with type 2 diabetes. Baseline 25-OH vitamin D was estimated by the following two ways: 1) quartiles (the second quartile as the reference group); 2) four groups (deficiency <25 nmol/L; insufficiency 25–49 nmol/L; sufficiency 50–99 nmol/L (reference group); and high vitamin D concentrations >100 nmol/L). We chose the second quartile of 25-OH vitamin D or 25-OH vitamin D sufficiency 50–99 nmol/L as the reference because these two groups had the lowest HRs of mortality in the restricted cubic spline, or according to the recommendations of the Institute of Medicine (18) or the Endocrine Society (8). Different levels of 25-OH vitamin D were included as dummy and categorical variables in the models, and the significance of the nonlinearity over different groups of 25-OH vitamin D concentrations was tested by giving an ordinal numeric value in the same models for each dummy variable. All analyses were multivariable-adjusted for age and sex, and further adjusted for duration of diabetes, alcohol drinking, smoking, family history of cardiovascular disease (CVD), insurance status, LDL cholesterol, eGFR, HbA1c, BMI, and use of anti-hypertensive drugs, anti-platelet agents, cholesterol-lowering agents, and glucose-lowering agents. To assess whether there was a dose–response or non-linear relationship between the circulating 25-OH vitamin D level as a continuous variable and all-cause mortality, the analysis was performed by the restricted cubic spline nested in Cox hazard regression model. The results were presented as a smoothed plot of hazard ratios (HRs) and 95% Confidence Intervals (CIs) for all-cause mortality. Kaplan–Meier analysis was performed to estimate the association between circulating 25-OH vitamin D concentrations and all-cause mortality among patients with type 2 diabetes. SPSS Statistics 25.0 software (IBM SPSS, Chicago, IL) and SAS for Windows, version 9.4 (SAS Institute, Inc, Cary, NC) were used to perform the analyses.

## Results

Basic characteristics of the participants are presented in **Tables 1**, **2**. During a median follow-up of 4.15 years (5,365 person-years in total), 61 patients died. Patients who died were older, had a longer duration of diabetes, were less likely to be obese, had higher HbA1c levels and higher 25-OH vitamin D levels compared with patients who lived. Multivariable-adjusted (age, sex, duration of diabetes, insurance status, smoking, alcohol drinking, systolic blood pressure, HbA1c, LDL cholesterol, eGFR, history of CVD, use of anti-hypertensive drugs, anti-platelet agents, cholesterol-lowering agents and glucose-lowering agents—Model 3) HRs for all-cause mortality across quartiles of baseline 25-OH vitamin D were 2.70 (95% CI 1.12–6.54), 1.00, 1.39 (95% CI 0.53–3.65), 2.31 (95% CI 0.96–5.54), respectively (**Table 3** and **Figure 2**). Multivariable-adjusted HRs for all-cause mortality based on different concentrations of circulating 25-OH vitamin D (<25, 25–49, 50–100, and ≥100 nmol/L) were 1.31 (95% CI 0.58–2.96), 0.94 (95% CI 0.47–1.87), 1.00, and 3.58 (95% CI 1.43–8.98), respectively (**Table 4**).

**Table 1:** Baseline characteristics of the study participants according to quartiles of 25-OH vitamin D.

	Quartiles of 25-OH Vitamin D				*P*-value
	1	2	3	4	
No. of participants	323	322	323	323	
Age, years	57.3 ± 15.3	56.5 ± 3.8	55.8 ± 4.5	59.2 ± 43.3	0.017
Female, n (%)	196 (60.7)	173 (53.7)	184 (57.0)	182 (56.3)	0.355
Body mass index, kg/m^2^	27.0 ± 4.9	26.8 ± 4.3	26.5 ± 44.2	25.8 ± 44.3	0.004
Duration of diabetes, years	9.81 ± 8.29	8.93 ± 7.82	9.34 ± 7.77	10.3 ± 7.7	0.155
25-OH Vitamin D, nmol/L	22.8 ± 3.7	32.7 ± 2.9	43.5 ± 3.7	78.8 ± 47.2	<0.001
25-OH Vitamin D, ng/ml	9.1 ± 1.5	13.1 ± 1.2	17.4 ± 1.5	31.5 ± 18.9	<0.001
Systolic blood pressure, mmHg	137 ± 20	135 ± 19	134 ± 19	135 ± 19	0.188
Diastolic blood pressure, mmHg	81 ± 11	81 ± 10	80 ± 11	80 ± 11	0.783
HbA_1c_, %	8.62 ± 2.14	8.35 ± 2.05	8.44 ± 2.07	8.05 ± 1.96	0.005
LDL cholesterol, mmol/L	3.16 ± 1.49	3.01 ± 1.09	3.09 ± 1.04	2.89 ± 1.03	0.023
Health insurance, n (%)	297 (92.0)	288 (89.4)	289 (89.5)	297 (92.0)	0.497
Current smoking, n (%)	88 (27.2)	88 (27.3)	96 (29.7)	95 (29.4)	0.842
Current alcohol drinker, n (%)	54 (16.7)	67 (20.8)	54 (16.7)	76 (23.5)	0.076
Use of medications, n (%)					
Anti-hypertensive	171 (52.9)	156 (48.4)	145 (44.9)	181(56.0)	0.025
Lipid-lowering	155 (48.0)	154 (47.8)	151 (46.7)	152 (47.1)	0.987
Anti-platelet	91 (28.2)	67 (20.8)	65 (20.1)	72 (22.3)	0.061
Glucose-lowering	319 (98.8)	320 (99.4)	318 (98.5)	315 (97.5)	0.262
Oral	292 (90.4)	304 (94.4)	306 (94.7)	298 (92.3)	0.109
Insulin	248 (76.8)	238 (73.9)	229 (70.9)	250 (77.4)	0.207

HbA_1c_, glycated hemoglobin A1c; LDL cholesterol, low-density lipoprotein cholesterol.

**Table 2:** Baseline characteristics of the study participants according to primary outcome.

	Primary Outcome		*P*-value
	Death	No Death	
No. of participants	61	1,230	
Female, n (%)	29 (47.5)	706 (57.0)	0.145
Age, years	68.7 ± 11.4	56.6 ± 14.2	<0.001
Body mass index, kg/m^2^	25.4 ± 4.1	26.6 ± 4.5	0.049
Duration of diabetes, years	13.5 ± 9.65	9.40 ± 7.77	<0.001
25-OH vitamin D, nmol/L	63.8 ± 47.3	43.9 ± 27.3	<0.001
25-OH vitamin D, ng/ml	25.5 ± 18.9	17.7 ± 10.9	<0.001
Systolic blood pressure, mmHg	136 ± 21	135 ± 19	0.519
Diastolic blood pressure, mmHg	81 ± 10	81 ± 10	0.516
HbA_1c_, %	8.74 ± 2.09	8.33 ± 2.04	0.138
LDL cholesterol, mmol/L	2.97 ± 1.09	3.03 ± 1.19	0.717
Health insurance, n (%)	57 (93.4)	1,114 (90.6)	0.650
Current smoking, n (%)	19 (31.1)	348 (28.3)	0.663
Current alcohol drinker, n (%)	11 (18.0)	240 (19.5)	0.869
Use of medications, n (%)			
Anti-hypertensive	37 (60.7)	616 (50.1)	0.069
Lipid-lowering	23 (37.7)	589 (47.9)	0.077
Anti-platelet	20 (32.8)	275 (22.4)	0.062
Glucose-lowering			
Oral	54 (88.5)	1,146 (93.2)	0.132
Insulin	51 (83.6)	914 (74.3)	0.130

HbA_1c_, glycated hemoglobin A1c; LDL cholesterol, low-density lipoprotein cholesterol.

**Table 3:** Hazard ratios of all-cause mortality by quartiles of 25-OH vitamin D levels among patients with type 2 diabetes.

25-OH Vitamin D(nmol/L)	No. of Participants	No. of Death	Pearson-Years	Hazard Ratios (95% Confidence Intervals)			
				Model 1	Model 2	Model 3	Model 4
Quartile 1	323	22	1,276	2.79 (1.18–6.56)	2.82 (1.19–6.66)	2.70 (1.12–6.54)	2.72 (1.12–6.60)
Quartile 2	322	7	1,281	1.00	1.00	1.00	1.00
Quartile 3	323	11	1,334	1.47 (0.57–3.79)	1.46 (0.57–3.78)	1.39 (0.53–3.65)	1.40 (0.53–3.67)
Quartile 4	323	21	1,474	2.34 (0.99–5.52)	2.38 (1.00–5.64)	2.31 (0.96–5.54)	2.17 (0.90–5.21)

Model 1 adjusted for age and sex; Model 2 adjusted for age, sex, insurance status, smoking, and alcohol drinking; Model 3 adjusted for age, sex, insurance status, smoking, alcohol drinking, duration of diabetes, systolic blood pressure, HbA1c, eGFR, LDL cholesterol, history of CVD, use of anti-platelet agents, anti-hypertensive drugs, glucose-lowering agents, and cholesterol-lowering agents statins; Model 4 adjusted for adjusted for age, sex, insurance status, smoking, alcohol drinking, duration of diabetes, systolic blood pressure, HbA1c, eGFR, LDL cholesterol, history of CVD, use of anti-platelet agents, anti-hypertensive drugs, glucose-lowering agents, cholesterol-lowering agents statin, and BMI.

Cut-points of quartile were 28.1, 37.8, and 50.7 nmol/L.

**Figure 2:** Multivariate-adjusted cumulative survival curves of all-cause mortality by different levels of 25-OH vitamin D levels. Adjusted for age, sex, insurance status, smoking, and alcohol drinking.

**Table 4:** Hazard ratios of all-cause mortality by different levels of 25-OH vitamin D levels among patients with type 2 diabetes.

25-OH Vitamin D (nmol/L)	No. of Participants	No. of Death	Pearson-Years	Hazard Ratios (95% Confidence Intervals)			
				Model 1	Model 2	Model 3	Model 4
<25	214	13	851	1.28 (0.59–2.79)	1.29 (0.59–2.80)	1.31 (0.58–2.96)	1.34 (0.59–3.05)
25–49	741	27	2,981	0.97 (0.50–1.89)	0.95 (0.49–1.85)	0.94 (0.47–1.87)	0.98 (0.49–1.95)
50–100	289	13	1,305	1.00	1.00	1.00	1.00
>100	47	8	229	2.90 (1.20–7.01)	3.01(1.23–7.34)	3.58 (1.43–8.98)	3.41 (1.35–8.61)

Model 1 adjusted for age and sex; Model 2 adjusted for age, sex, insurance status, smoking, and alcohol drinking; Model 3 adjusted for age, sex, insurance status, smoking, alcohol drinking, duration of diabetes, systolic blood pressure, HbA1c, eGFR, LDL cholesterol, history of CVD, use of anti-platelet agents, anti-hypertensive drugs, glucose-lowering agents, and cholesterol-lowering agents statins; Model 4 adjusted for adjusted for age, sex, insurance status, smoking, alcohol drinking, duration of diabetes, systolic blood pressure, HbA1c, eGFR, LDL cholesterol, history of CVD, use of anti-platelet agents, anti-hypertensive drugs, glucose-lowering agents, cholesterol-lowering agents statin, and BMI.

Multivariable-adjusted (Model 3) HRs for all-cause mortality across quartiles of baseline 25-OH vitamin D were 4.45 (95% CI 1.16–17.1), 1.00, 1.30 (95% CI 0.28–6.14), 2.90 (95% CI 0.72–11.7) for men, and 2.68 (95% CI 1.26–10.7), 1.00, 1.54 (95% CI 0.34–7.10), 2.42 (95% CI 0.62–9.44) for women, respectively.

When baseline circulating 25-OH vitamin D was examined as a continuous variable by using restricted cubic splines, a nadir of a U-shaped association of baseline circulating 25-OH vitamin D with all-cause mortality was observed at a 25-OH vitamin D level of 33 nmol/L (**Figure 3**).

**Figure 3:** Adjusted hazard ratios (solid line) and 95% confidence interval (dashed lines) for all-cause mortality according to different levels of 25-OH vitamin D. Adjusted for age, sex, insurance status, smoking, and alcohol drinking.

## Discussion

The present study found a U-shaped association of baseline 25-OH vitamin D levels with all-cause mortality risk among patients with type 2 diabetes. An increased risk of all-cause mortality was observed among patients with very low or high concentrations of 25-OH vitamin D.

Vitamin D exhibits an extensive range of biological functions, namely, anti-inflammatory, inhibiting cellular proliferation, prodifferentiative, antioxidative, and immunomodulatory effects (21, 22), which implies that vitamin D deficiency might be associated with various pathological conditions and proper supplementation of vitamin D could translate into health benefits (23, 24). Epidemiological evidence reveals that severe vitamin D deficiency is a risk factor for multiple adverse health outcomes, such as cause-specific mortality and all-cause mortality (25–27). A prior study indicated that an inverse relationship between vitamin D status and all-cause mortality only existed in individuals with vitamin D insufficiency or deficiency (28). Several clinical randomized trials did not find any benefits of vitamin D supplementation for the prevention of cardiovascular disease or mortality (29, 30). For instance, the Vitamin D and Omega-3 Trial (VITAL) (31) indicated that vitamin D supplements did not decrease the incidence of cardiovascular and invasive cancer events compared with placebo. A meta-analysis involving 74,655 participants also revealed that supplementation of vitamin D alone was not associated with the risks of all-cause or cause-specific mortality among adults (24). Thus, the effect of vitamin D supplementation on mortality and the relationship between circulating Vitamin D concentrations and all-cause mortality need further elucidation.

As mentioned above, many studies have focused on the effects of vitamin D deficiency and the potential benefits of vitamin D supplementation. Only a few studies have examined the associations between high vitamin D concentrations and the risk of all-cause mortality. Emerging epidemiological evidence indicates that there is a non-linear relationship between baseline circulating 25-OH vitamin D levels and all-cause mortality (12). An investigation-COPD study in Denmark (32) illustrated that a concentration of vitamin D over 140 nmol/L or a very low concentration of vitamin D might increase all-cause mortality risk among the general population. The NHANES III study (1988–1994) suggested a reverse J-shaped association between serum 25-OH vitamin D levels and the 9-year risk of all-cause mortality (33). Moreover, after additional 6-year follow-up, the reverse J-shaped association persisted through 15 years of follow-up, with a strong inverse association when 25-OH vitamin D was below 40 nmol/L, and with a weak increased risk when 25-OH vitamin D was over 120 nmol/L (15). A previous cohort study involving a total of 24,094 inpatients in Boston revealed that 25-OH vitamin D levels less than 20 ng/ml or over 60 ng/ml before hospitalization were associated with an increased odds of 90-day mortality (34). However, the population from above studies did not include patients with type 2 diabetes. Only a few studies have focused on the relationship between baseline circulating vitamin D levels and all-cause mortality among patients with type 2 diabetes. The cohort analysis from the NHANES III and the NHANES 2001–2014 involving 6,329 patients with type 2 diabetes indicated that the multivariate-adjusted HR of all-cause mortality for individuals with 25-OH vitamin D >75 nmol/L was 0.59 (95% CI 0.43–0.83) compared with subjects with 25-OH vitamin D <25 nmol/L (11). Another analysis from the NHANES III and the NHANES 2001–2014 involving 15,195 patients with prediabetes suggested that per unit increase in ln-transformed 25-OH vitamin D was associated with a 27% lower risk of all-cause mortality (35). Whereas, in the present study, compared with vitamin D sufficient persons (50–100 nmol/L), all-cause mortality risk was significantly higher among type 2 diabetic patients with both low baseline vitamin D level and high concentrations of over 100 nmol/L. The discrepancy between the NHANES cohort study and the present study could be explained by diverse populations with different races and observational cohort studies are susceptible to uncontrolled confounding factors, such as dietary intake factors, physical activity and sunlight time. Since above studies were observational in nature, such that casual associations between either low or high circulating 25-OH vitamin D levels and higher mortality could not be ascertained, supplementation with vitamin D among people with type 2 diabetes should be evaluated carefully.

Although the mechanism of how vitamin D deficiency increased the all-cause mortality risk is not completely clear. Growing evidence has shown that vitamin D has an extensive noncalcemic pleiotropic function mediated by vitamin D receptor (VDR) (36), associated with suppression of the renin-angiotensin system (37), anti-myocyte hypertrophy (38), atherosclerosis lowering (39, 40) and anti-inflammation (41, 42). The activation of VDR in cardiomyocytes and endothelial cells could regulate vascular tension and smooth muscle contractions, thus providing protective effect on endothelial dysfunction (43). Moreover, some studies indicated that vitamin D could affect pancreatic endocrine function (44), resulting in impaired glucose metabolism and insulin resistance among subjects with low vitamin D levels (45, 46). In view of the extensive biological functions of vitamin D (47) and high probability of fracture caused by vitamin D deficiency, it is easy to accept that vitamin D deficiency might increase mortality. However, the effect of high concentrations of vitamin D on all-cause mortality is still under debate and the findings that high concentrations of vitamin D were associated with an increased risk of mortality seemed paradoxical. Several putative mechanisms may be proposed: First, there might be interaction between disease status and 25-OH vitamin D levels. Poor health status might lead to vitamin D deficiency. As the increasing media reported on the demand to take enough vitamin D, subjects with illness or poor health were supposed to have extra vitamin D supplemented after disease development, which might result in a U-shaped or J-shaped association between vitamin D concentrations and the risk of all-cause mortality. The Uppsala health survey in Sweden involving 1,194 adult men demonstrated a U-shaped association between vitamin D levels and all-cause mortality when prior disease status was adjusted for, or persons with cardiovascular disease or cancer at baseline were excluded (14). The all-cause mortality risk was 1.5–1.6 fold higher in the lowest 10% and the highest 5% of the plasma 25-OH vitamin D distributions (14). Second, some experimental studies showed that excessive vitamin D might accelerate aging (48) and promote cancer through the stimulatory effects of vitamin D on enzyme CYP24 and insulin-like growth factor I (IGF-I) production (49). Moreover, along with the increased awareness of vitamin D supplementation, extra intake higher than the upper limit may increase the incidence of vitamin D toxicity (50).

Our study has several strengths. First and foremost, the present study is a cohort study rather than a cross-sectional study, thus providing an accurate and comprehensive analysis. A recent literature review (51) has summarized published articles on the potential effects of medication such as glucose-lowering agents, anti-hypertensive drugs, and cholesterol-lowering agents on the vitamin D concentration. Thus, the other important advantage of our study is that some potential factors, such as glucose-lowering agents, anti-hypertensive drugs, and cholesterol-lowering agents which could affect the vitamin D level, were taken into consideration. The present study also has some limitations. First, the study sample from a single clinical center was relatively small, which limited the generalizability. Second, 25-OH vitamin D was measured only once at baseline. Changes in 25-OH vitamin D levels might be associated with all-cause mortality risk. Third, some residual confounding factors such as physical activity, sunlight time and dietary factors, which are associated with vitamin D levels, have not been included, even though our analyses adjusted for major confounding variables. Fourth, the 25-OH vitamin D assay was not accredited by the Vitamin D External Quality Assessment Scheme (DEQAS), which limited the precision. Fifth, due to the limited sample size, sensitivity analyses were not made completely. Last, withdraw bias might be induced because some patients could not be reached by telephone follow-up or unwilling to tell us the information about the patients, and death was documented by telephone follow-up, rather than linked death registry.

In conclusion, the present study found a U-shaped association of baseline 25-OH vitamin D levels with all-cause mortality risk among patients with type 2 diabetes. An increased risk of all-cause mortality was observed among patients with very low or high concentrations of 25-OH vitamin D. Direct experimental investigation and large randomized clinical trials are still necessary to identify the precise curve and whether supplementation of vitamin D could reduce all-cause mortality among either specific populations or general populations.

## Data Availability Statement

Data described in this article, the code book, and the analytic code will be made available upon request.

## Ethics Statement

The study was approved by the Tianjin Medical University General Hospital Institutional Review Board with waiver of individual informed consent (approval number IRB2020-YX-027-01). Written informed consent for participation was not required for this study in accordance with the national legislation and the institutional requirements.

## Author Contributions

Y.Z, H.S., and L.D. researched the data. Y.F. and L.D. wrote the manuscript. Q.H., J.C. and G.H reviewed and revised the manuscript. M.L. had full access to all the data in the study and took responsibility for the integrity of the data and the accuracy of the data analysis. All authors listed have made a substantial, direct, and intellectual contribution to the work and approved it for publication.

## Funding

This work was supported by research grants from the National Natural Science Foundation for Young Scholars of China 81800733.

## Conflict of Interest

The authors declare that the research was conducted in the absence of any commercial or financial relationships that could be construed as a potential conflict of interest.

## Publisher’s Note

All claims expressed in this article are solely those of the authors and do not necessarily represent those of their affiliated organizations, or those of the publisher, the editors and the reviewers. Any product that may be evaluated in this article, or claim that may be made by its manufacturer, is not guaranteed or endorsed by the publisher.
